RETRACTED

# Transglutaminase is a mesothelioma cancer stem cell survival protein that is required for tumor formation

**DOI:** 10.18632/oncotarget.26130

**Published:** 2018-10-02

**Authors:** Gautam Adhikary, Daniel Grun, H. Richard Alexander, Joseph S. Friedberg, Wen Xu, Jeffrey W. Keillor, Sivaveera Kandasamy, Richard L. Eckert

**Affiliations:** ^1^ Departments of Biochemistry and Molecular Biology, University of Maryland School of Medicine, Baltimore, Maryland, USA; ^2^ Department of Dermatology, University of Maryland School of Medicine, Baltimore, Maryland, USA; ^3^ Department of Reproductive Biology, University of Maryland School of Medicine, Baltimore, Maryland, USA; ^4^ Greenebaum Comprehensive Cancer Center, University of Maryland School of Medicine, Baltimore, Maryland, USA; ^5^ Department of Surgery and Division of General and Surgical Oncology, University of Maryland School of Medicine, Baltimore, Maryland, USA; ^6^ Department of Chemistry, University of Ottawa, Ottawa, ON, CA; ^7^ Department of Surgery, Rutgers Robert Wood Johnson Medical School, New Brunswick, New Jersey, USA

**Keywords:** mesothelioma, transglutaminase, TGM2, cancer stem cell, EMT

## Abstract

Mesothelioma is a rare cancer of the mesothelial cell layer of the pleura, peritoneum, pericardium and tunica vaginalis. It is typically caused by asbestos, notoriously resistant to chemotherapy and generally considered incurable with a poor life expectancy. Transglutaminase 2 (TG2), a GTP binding regulatory protein, is an important cancer stem cell survival and therapy resistance factor. We show that TG2 is highly expressed in human mesothelioma tumors and in mesothelioma cancer stem cells (MCS cells). TG2 knockdown or TG2 inhibitor treatment reduces MCS cell spheroid formation, matrigel invasion, migration and tumor formation. Time to tumor first appearance is doubled in TG2 knockout cells as compared to wild-type. In addition, TG2 loss is associated with reduced expression of stemness, and epithelial mesenchymal transition markers, and enhanced apoptosis. These studies indicate that TG2 is an important MCS cell survival protein and suggest that TG2 may serve as a mesothelioma cancer stem cell therapy target.

## INTRODUCTION

Mesothelioma is a primary cancer of the mesothelial cell layer of the pleura, peritoneum, pericardium or tunica vaginalis. It is generally considered incurable and often portends a poor life expectancy [1, 2]. Mesothelioma is typically caused by exposure to asbestos or, less commonly, presents as a secondary malignancy related to radiation [1, 2]. Due to the “coating nature” of mesothelioma it is not possible to achieve a microscopically complete resection and is, consequently, not considered curable with surgery. The standard of care treatment for most presentations of mesothelioma is chemotherapy alone, but mesothelioma is a notoriously drug-resistant disease [2]. The response rate for chemotherapy when mesothelioma occurs in the chest, for instance, is approximately forty percent [3]. This clinical experience speaks to the need for new therapeutic approaches.

RETRACTED

We hypothesize that mesothelioma cancer stem (MCS) cells survive tumor excision/chemotherapy and give rise to drug-resistant cells that drive aggressive tumor regrowth. We further propose that effective therapies must target these cells. Our approach, in this context, is to identify proteins that are essential for MCS cell survival and then eliminate or inactivate these proteins to reduce survival. Working towards this goal, we developed systems for propagation of human MCS cells [4]. These cells display properties of cancer stem cells including self-renew and high level expression of stem cell markers [4].

Of particular importance, we now show that tissue transglutaminase (TG2), a GTP binding signaling protein and regulator of cancer stem cell survival [5–8], is highly enriched in MCS cells compared to non-stem cancer cells. TG2 is a unique member of the transglutaminase family that has received considerable attention relating to its newly-discovered role as a regulator of stem cell function [9–12]. Intracellular TG2 exists in a closed conformation and functions as GTP binding signaling protein that is intimately involved in cell survival signaling [5–9, 13]. TG2 level is markedly increased in tumors and tumor cell lines [14–18] and expression is associated with increased metastasis and drug resistance [19–23]. At a functional level, TG2 drives survival signaling, reduces expression of tumor suppressor genes, drives synthesis and deposition of fibronectin and collagen, and stimulates epithelial-mesenchymal transition (EMT) [18, 24]. In addition, TG2 has an important role in cancer cell acquisition of cancer stem-cell traits [7, 8, 25–27]. Elevated TG2 expression is associated with enhanced cancer stem cell survival and resistance to chemotherapy [28] and knockdown of TG2 results in re-sensitization of cancer cells to conventional anti-cancer drugs [28]. This is important, as treatment with conventional drugs can select for TG2-enriched cells [25, 29].

In the present study, we examine the role of TG2 as a survival factor in mesothelioma. We show that TG2 is highly enriched in mesothelioma as compared to normal mesenchymal tissue, and is highly elevated in MCS cells as compared to non-stem cancer cells. In addition, TG2 knockout or treatment with a TG2-specific inhibitor reduces spheroid formation, matrigel invasion, migration and tumor formation.

RETRACTED

## RESULTS

### TG2 is required for the MCS cell phenotype

We first confirmed that cancer stem cell-enriched spheroid can be formed by Meso-1 cells [4]. Figure 1A compares the growth of monolayer and spheroid cultures. Only a small percentage (0.15%) of monolayer cells plated in spheroid growth conditions survive beyond 12–24 h and form spheroids. This suggests that only 0.15% of the cancer cells manifest an intrinsic mesothelioma cancer stem (MCS) cell phenotype. Figure 1B shows that spheroid number and size increase progressively with time in culture. Biochemical analysis indicates that MCS cells (spheroid-derived) express markedly elevated levels of TG2, as compared to non-stem (monolayer-derived) cancer cells (Figure 1C). Moreover, consistent with a potential role in disease pathogenesis, TG2 levels are markedly overexpressed in human tumors as compared to normal mesenchymal tissue (Figure 1C).

**Figure 1:** TG2 is enriched in MCS cells and required for survival (**A**, **B**) Meso-1 monolayer cells were harvested and seeded in ultra-low attachment plates for growth as spheroids (MCS cells). (**C**) TG2 level is markedly enriched in MCS cells and human tumors (T1/T2 = tumors, N1/N2 = control tissue). (**D**–**J**) TG2 is required for optimal cell proliferation, spheroid formation, invasion and migration. The values are mean ± SEM and the asterisks indicate a significant change compared to control, *n* = 3, *p* < 0.005. The bars = 50 microns in all panels.

To assess the role of TG2 in maintaining the MCS cell phenotype, we created TG2 knockout Meso-1 cells (Meso1-TG2-KOc4) (Figure 1D) and used these cells to study the role of TG2 in maintaining MSC cell survival. Figure 1E shows that Meso1-TG2-KOc4 cell monolayer cultures proliferate more slowly than wild-type cells. We next examined the impact of TG2 knockdown on cancer stem cell biological responses including spheroid formation, matrigel invasion and migration [11]. Figure 1F, 1G shows that TG2 null cells form reduced numbers of spheroids of smaller size. Moreover, these spheroids are abnormal in appearance and the cultures accumulate cell debris (Figure 1H). In addition, Meso1-TG2-KOc4 cells display reduced ability to invade matrigel and migrate on plastic to close a wound (Figure 1I, 1J).

### Elevated TG2 is associated with EMT

Enhanced cancer cell stemness is frequently associated with increased epithelial-mesenchymal transition (EMT) [8, 11, 25]. We therefore monitored the impact of TG2 on EMT. Figure 2A displays images of Meso-1 non-stem cancer cells (monolayer) and MCS cells (spheroid) cultures used for biochemical studies of EMT. Figure 2B shows that TG2 is increased in MCS cell cultures and that this is associated with an increase in selected EMT markers. Fibronectin, MMP-9, Slug and Snail levels are increased, but vimentin level is not changed and N-cadherin level is slightly decreased. We next compared TG2 and EMT marker levels in human tumor samples. Figure 2C shows a general increase in EMT markers in mesothelioma tumor samples (T1, T2) as compared to normal tissue (N1, N2). We also assayed for polycomb gene expression and activity. Polycomb proteins are often elevated in tumors where they modify histones to close chromatin and reduce tumor suppressor expression to accelerate tumor growth [30, 31]. Figure 2C shows that elevated TG2 expression in human mesothelioma tumors is associated with increased polycomb protein (Ezh2, Suz12 and Bmi-1) levels, and increased polycomb activity as evidence by increased H3K27me3 formation. TG2 appears to have a role in controlling EMT, as TG2 knockdown reduces fibronectin, Snail and Slug level (Figure 2D).

RETRACTED

**Figure 2:** TG2 expression is associated with enhanced EMT marker expression (**A**, **B**) Monolayer and spheroid cultures were grown for 8 d and extracts were prepared for detection of the indicated epitopes. (**C**) Extracts were prepared from normal human tissue (N1/N2) and tumors (T1/T2) for epitope detection by immunoblot. (**D**) Meso-1 and Meso-1-TG2-KOc4 cells were grown as spheroids and extract was prepared for detection of the indicated proteins. Similar results were observed in multiple experiments. Each experiment indicated in this figure were repeated a minimum of three times. Bars = 50 microns in all panels.

We next determined whether TG2 is required for MCS cell survival in another peritoneal-derived mesothelioma cell line, Meso-2. Meso-2 cells were electroporated with control- or TG2-siRNA and knockdown of TG2 was confirmed (Figure 3A). TG2 knockdown in Meso-2 cells is associated with reduced spheroid formation and spheroid size, as well as, accumulation of debris in the spheroid cultures (Figure 3B) and a reduction in matrigel invasion and wound closure-related migration (Figure 3C, 3D).

**Figure 3:** TG2 knockdown reduces MCS cell properties in Meso-2 cells (**A**) Meso-2 cells were treated with 3 µg of control- or TG2-siRNA and after 48 h extracts were prepared to monitored TG2 level. (**B**–**D**) TG2 knockdown in Meso-2 cells reduces spheroid number and size, matrigel invasion and migration. The values are mean ± SEM and asterisks indicate a significant change compared to control, *n* = 3, *p* < 0.05. Bars = 50 microns in all panels.

### NC9 inhibition of TG2 reduces MCS survival

Pharmacologic inhibition of TG2 is an important anti-cancer therapy option. We therefore determined if treatment with NC9, an efficient irreversible small molecule TG2 inhibitor [32, 33], suppresses the MCS cell phenotype. NC9 binds to the TG2 transamidase site to cause a TG2 conformation change that inactivates the TG2 transamidase and GTP binding activities [33]. NC9 treatment reduces Meso-1 (Figure 4A–4C) and Meso-2 (Figure 4E–4G) cell spheroid formation, invasion and migration. In addition, loss of TG2 reduces polycomb protein level (Ezh2, Bmi-1) and activity (H3K27me3) and stem cell marker (Sox-2, Oct-4) level. Apoptosis, as evidenced by increased caspase-9 and PARP activity, is also increased (Figure 4D, Figure 4H).

RETRACTED

**Figure 4:** NC9 treatment suppresses the MCS cell phenotype (**A**–**D**) Meso-1 cells were monitored for spheroid formation, invasion and migration, and expression of MCS cell-associated markers following treatment with 0, 50 and 100 µM NC9. (**E**–**H**) Meso-2 cells were monitored as described for Meso-1. The values are mean ± SEM and asterisks indicate a significant change compared to control, *n* = 3, *p* < 0.05. Bars = 50 microns in all panels.

### Role of TG2 in tumor formation

To assess the role of TG2 in tumor formation, we compared tumor growth of non-stem (monolayer) and MCS (spheroid) cells. MCS cells form rapidly growing and aggressive tumors (Figure 5A) that are enriched in TG2 and EMT markers (Figure 5B). Moreover, MCS cell-derived tumors appear more vascularized which is consistent with increased levels of the CD31, an endothelial cell-specific marker of vascularization (Figure 5C). To determine if TG2 impacts tumor formation, we compared tumor growth for TG2-positive and negative Meso-1 cells. Figure 5D shows that TG2-positive MCS cell tumors appear at 9 wk, while appearance of TG2-null cells tumors is delayed until 18 wk. Moreover, TG2-positive tumors are nearly 400 cubic millimeters at 16 wks, but TG2-negative cell tumors are not yet detected. Figure 5E provides evidence that TG2 knockdown reduces EMT marker (Fibronectin, Slug, Snail and Twist) levels in tumors, but that other markers are not substantially altered. However, we were surprised to observe TG2 in extracts from TG2 knockout cell-derived tumors. This could be contamination from surrounding cell types or TG2 re-expression in the knockout tumor cells. We therefore cultured cells from TG2 wild-type and TG2 knockout tumors and monitored TG2 level. Figure 5F shows that cells from the knockout tumors lack TG2 expression, thereby confirming the knockout status of the tumor cells.

**Figure 5:** TG2 is required for optimal tumor formation (**A**–**C**) Monolayer- and spheroid-derived Meso-1 cells were injected (3 million/injection) into each front flank in NSG mice and tumor formation was monitored. Extracts were prepared from 16 wks tumors for detection of the indicated epitopes. (**D**, **E**) Meso-1 and Meso1-TG2-KOc4 cells were grown as spheroids and tumor formation was monitored in NSG mice. Extracts were prepared from 16 wk Meso-1 cell and 21 wk Meso1-TG2-KOc4 cells for detection of the indicated epitopes. (**F**) Meso-1 and Meso1-TG2-KOc4 tumors were harvested and tumor cells were isolated and grown in culture for preparation of extracts to measure TG2 level. (**G**–**I**) Spheroid derived Meso-1 cells were injected at 3 million cells per each front flank in five NSG mice per treatment, and at 8 wks post-injection treatment was initiated with the indicated levels of NC9. Tumor growth was monitored and at 14 wks images were collected and extracts prepared to monitor the impact of NC9 treatment on the indicated epitopes. Similar results were observed in multiple experiments. The values are mean ± SEM and the asterisks indicate a significant change compared to control, *n* = 3 experiments, *p* < 0.05. (**J**) A schematic of TG2 impact on MSC cell phenotype. TG2 increases the indicated processes and this can be inhibited by the TG2 inhibitor, NC9.

RETRACTED

We next determined if NC9 can suppress MCS cell tumor formation. Meso-1 cells were injected into each front flank in NSG mice and after eight wks NC9 treatment was initiated. NC9 treatment produces a marked reduction in tumor formation (Figure 5G, 5H) and this is associated with a parallel reduction in stem cell (Sox-2, Oct-4) and EMT (fibronectin, N-cadherin, Slug and Twist) marker levels (Figure 5I).

## DISCUSSION

Mesothelioma is one of the most virulent and treatment resistant cancers known to man, considered incurable and often with survival cited in the one year range. Palliative chemotherapy, with a poor response rate, is currently the standard of care in the United States for the majority of mesothelioma patients. This standard treatment has not changed for over a decade. Thus, there is a pressing need for new treatments for this cancer. Cancer stem cells have been identified in mesothelioma [4, 34, 35] and in other cancers [10, 36]. These cells are highly aggressive tumor-forming cells as compared to non-stem cancer cells. It is thought that cancer stem cells give rise to daughter cells that populate tumors and that targeting stem cells for treatment is a productive strategy to reduce tumor growth. For this reason, we have focused on identifying proteins/activities that are elevated in cancer stem cells and facilitate cancer stem cell survival [10, 11, 36]. TG2 expression is associated with formation of highly aggressive cancers [7, 10, 12, 26, 27, 37, 38] and is enriched in cancer stem cells [10, 39].

RETRACTED

### TG2 maintains the MCS cell phenotype

In the present report, we show that TG2 level is elevated in human mesothelioma tumors, and is enriched in MCS cells as compared to non-stem cancer cells. We further show that TG2 is required to maintain activities that are enhanced in MCS cells including spheroid formation, invasion and migration. TG2 knockout cells display much reduced spheroid formation, invasion and migration. At the biochemical level, increased TG2 in human mesothelioma tumors and in MSC cells is associated with enhanced expression of polycomb group and EMT proteins. The polycomb proteins are epigenetic regulators that methylate histones to silence expression tumor suppressor gene expression and enhance cell survival [40, 41]. Previous studies show that polycomb proteins enhance cancer cell survival and tumor formation [42, 43]. Tumors and MCS cells display elevated expression of proteins involved in EMT, including Snail, Slug, N-cadherin and fibronectin, and TG2 knockdown reduces the level of these proteins. These findings are consistent with a role for TG2 in enhancing MCS cell EMT, as measured by enhance invasion and migration, and also with TG2 as a hypoxia response factor [44].

### TG2 inhibitor suppresses the MCS cell phenotype

An important goal is identification of agents that can selective target cancer stem cells in tumors. In this context, we tested a novel TG2 inhibitor, NC9, for ability to suppress the MCS cell phenotype. TG2 displays both transamidase and GTP binding activities, and NC9 covalently binds to TG2 to inactivate both of these activities [33, 45, 46]. NC9 treatment reduces polycomb group, cancer stem and EMT protein levels in MCS cells, and also increases caspase and PARP-associated apoptosis. This is observed in both Meso-1 and Meso-2 cells, suggesting it is a generalized response to TG2 inhibition, and is associated with a reduction in spheroid formation, invasion and migration. Thus, inhibition of TG2 markedly reduces processes associated with the aggressive MCS cell phenotype that are required for MCS cell survival, and also induces cell death.

### Role of TG2 in tumor formation

Growth as spheroids is an extremely useful method for selection of cells with cancer stem properties. When mesothelioma cells are cultured in this model, only 0.15% of cells survive to form spheroids. A comparison of tumor properties reveals that MCS cells, enriched by growth as spheroids, form substantially larger tumors and express higher levels of TG2 than non-stem mesothelioma cancer cells. These cells also express elevated stemness and EMT markers. We also examined the impact of TG2 knockdown on tumor formation. TG2-positive MCS cell tumors are first detected at week nine post-injection, but tumor appearance is delayed until week eighteen in TG2 knockout MSC cells. Thus, TG2 knockout doubles the time to first tumor appearance. In addition, the TG2 knockdown tumors express reduced levels of stem cell and EMT markers, and display reduced vascularity (i.e., reduced CD31 expression). Surprisingly, we found TG2 in extracts from TG2 knockout cell-derived tumors; however, we could not find TG2 when these cells were isolated from tumors and cultured, indicating that the TG2 is derived from other cell types in the tumor.

RETRACTED

As indicated in Figure 5J, our findings suggest that TG2 maintains the MCS cell phenotype [38, 47, 48], including enhancing spheroid growth, invasion and migration, angiogenesis, tumor growth, and EMT and stemness. We suggest that TG2 should be explored as a mesothelioma therapy target, as the MCS cell phenotype, including tumor formation, is markedly suppressed by treatment with the TG2-specific inhibitor, NC9.

## MATERIALS AND METHODS

### Antibodies and reagents

RPMI1640 medium (11875-093), sodium pyruvate, L-glutamine (25030-164), penicillin-streptomycin solution (15140-122) and 0.25% trypsin-EDTA (25200-056) were purchased from Gibco (Grand Island, NY). Antibodies for Ezh2 (612667), fibronectin (610077), N-cadherin (610920), PARP (556494) were obtained from BD transduction laboratories (San Jose, CA). H3K27me3 (07-449) and TG2 (MAB3839) antibodies were purchased from EMD Millipore (Bedford, MA). Antibodies for Bmi-1 (ab14389), Slug (ab27568), Twist (ab49254), HIF1-α (ab113642) and MMP9 (ab38898) were obtained from Abcam (Cambridge, UK). β-actin (A5441) antibody, heat inactivated fetal calf serum (FCS, F4135) and DAPI (D9542) were purchased from Sigma (St Louis, MO). Antibodies for vimentin (5741), cleaved PARP (9541), caspase-3 (9662), Snail (3895), p21Cip1 (2947), cleaved caspase-9 (9502) and Sox-2 (2748) were purchased from Cell Signaling Technologies (Danvers, MA). Peroxidase-conjugated anti mouse IgG (NXA931) and anti- rabbit IgG (NA934V) were obtained from GE Healthcare (Buckinghamshire, UK) and used at 1:5000 dilution. TG2- (sc-37514) and control-siRNA (sc-37007) and anti-Oct-4 (sc-9081) were purchased from Santa Cruz (Dallas, TX). Matrigel gel (354234) and BD BioCoat Millicell inserts (353097) were purchased from BD Bioscience (Franklin Lakes, NJ). The TG2 small molecule inhibitor, NC9, was prepared as previously described [45].

### Immunoblot

Cell or tumor samples were lysed in modified Laemmli buffer (0.063 M Tris-HCl, pH 7.5, 10% glycerol, 5% SDS, 5% β-mercaptoethanol) and equivalent amounts of protein were electrophoresed on denaturing and reducing 8% polyacrylamide gels and transferred to nitrocellulose membrane. The membrane was blocked by 5% non-fat dry milk and then incubated with the appropriate primary (1:1000) and then with secondary antibodies (1:5000). Secondary antibody binding was visualized using chemiluminescence detection technology.

RETRACTED

### Spheroid formation assay

Meso-1 and Meso-2 cells were maintained in RPMI1640 growth medium containing 2 µM L-glutamine supplemented with 10% heat inactivated FCS. Meso-1 and Meso-2 are immortal mesothelioma cell lines generated from malignant peritoneal mesothelioma solid tumor samples [49]. Eighty percent confluent cultures were dissociated with trypsin followed by serum-dependent trypsin inactivation. The cells were collected by centrifugation, re-suspended in RPMI1640 media supplemented with 10% FCS and grown as spheroids by platting 20,000 cells per 9.5 cm^2^ well with 3 ml medium in 6 well ultra-low attachment Costar cluster dishes (#4371, Corning, Tewksbury, MA). Parallel cultures were plated in the same growth medium on conventional plastic dishes for growth as monolayers. Cell culture medium was not changed during the experiment. We define a spheroid as a collection of cells achieving a diameter ≥ 25 µM. We counted the total number of spheroids in each of three dishes per group in each of three experiments and the values are plotted as mean ± SEM. Significant difference was assessed using the Student’s *t*-test.

### Meso-1 TG2 knockout cells

CRISPR/Cas9-based TG2 gene knockout plasmids purchased from Biocytogen (Worcester, MA). Meso-1 cells (1 million) were co-electroporated with 3 μg of plasmid and allowed to recover for 72 h. This process was repeated and after 72 h the cells were grown as monolayer cultures in fresh medium containing 1 μg/ml puromycin. The cells were passaged at 80% confluence in the presence of 1 μg/ml puromycin for 2 wk and single cells were collected for clonal expansion in the presence of puromycin. This produced clonal TG2 knockout cell lines, including Meso-1-TG2-KOc4. The TG2-null status of the clonal lines was confirmed by immunoblot.

### Cell invasion and migration assays

To measure cell invasion, BioCoat Millicell insert (1 cm diameter, 8 μm pore size) were coated with 120 µl of 250 μg/ml Matrigel. Cells (25,000) were seeded atop the matrigel in 500 μl of serum-free RPMI1640 containing 1% FCS. The lower chamber contained the identical medium containing 10% FCS. When appropriate, pharmacologic agents were added to the bottom chamber and the cells were placed in an incubator. After 18 h the membrane was washed, fixed with 4% paraformaldehyde and cells on the membrane inner surface were visualized by staining with 4’, 6-diamidino-2-phenylindole (DAPI) for fluorescence detection of nuclei. For the migration assay, confluent monolayer cultures were wounded by scraping with a 10 μl pipette tip and the released cells were removed. Migration of cells to close the wound was monitored at 0–18 h.

RETRACTED

### Tumor xenograft growth assays

Three million non-stem cancer cells (monolayer) or MCS cells (spheroid) were suspended in 100 μl phosphate buffered saline containing 30% matrigel followed by subcutaneous injection into the two front flanks of NOD *scid* IL2 receptor gamma chain knockout mice (NSG) using a 26.5 gauge needle. Five mice were used per treatment group. Tumor growth was monitored by measuring tumor diameter and calculating tumor volume = 4/3π × (diameter/2)^3^. For small molecular inhibitor studies, 3 million cells were injected into each front flank, and after 8 wks, when tumors were first palpable, inhibitor treatment was initiated by IP injection at final concentrations of 0, 20 and 50 mg/kg three times per week (M/W/F). A 0.3 M NC9 stock was prepared in DMSO and diluted into captisol at 2 and 4 mg/ml and 0.2 ml was IP injected per treatment for a final treatment concentration of 20 and 50 mg/kg body weight. NC9 treatment was initiated at the time tumors were detected at eight weeks post-injection. These studies were approved by the institutional board and followed accepted international practices for the treatment and welfare of animals.
